# Adverse Events following Immunization with COVID-19 Vaccines: A Narrative Review

**DOI:** 10.1155/2022/2911333

**Published:** 2022-08-16

**Authors:** Bijay Bhandari, Gaurav Rayamajhi, Pratik Lamichhane, Ashok K. Shenoy

**Affiliations:** ^1^Drug and Patient Safety Unit, Lumbini Provincial Hospital, Rupandehi, Nepal; ^2^Maharajgunj Medical Campus, Institute of Medicine, Tribhuvan University, Kathmandu, Nepal; ^3^Department of Pharmacology, Kasturba Medical College, Mangalore, Manipal Academy of Higher Education, Manipal, India

## Abstract

Numerous COVID-19 vaccines are being administered to people around the world. Adverse events following immunization (AEFI) with COVID-19 vaccines have been reported by health care workers as well as surveillance bodies. A wealth of information on the efficacy and safety of vaccines exists in the literature, and the knowledge in this sector is growing exponentially. A narrative literature review was conducted on sources accessed from PubMed, Google Scholar, and Cochrane Review from March 2021 to July 2021. This review is aimed at describing AEFI associated with currently available COVID-19 vaccines, with an emphasis on narrating probable AEFI, and at assisting in a better understanding of the COVID-19 vaccines.

## 1. Introduction

The Coronavirus Disease 2019 (COVID-19) pandemic has affected the entire globe. While it can take up to 10-14 years for a vaccine to be developed [1], many COVID-19 vaccines have emerged in this atypical period of high-speed clinical development. However, the expected vaccine outcome might overshadow the possible risks [2, 3]. The approval of COVID-19 vaccines is a major step in mitigating the devastating impact of COVID-19 [4]. Nevertheless, the vaccines might not be free from adverse effects that may remain undetectable in clinical trials, so evaluation, monitoring, and surveillance of adverse effects following immunization (AEFI) are vital [5, 6].

According to the World Health Organization (WHO), an AEFI is defined as “any untoward medical occurrence which follows immunization and which does not necessarily have a causal relationship with the usage of the vaccine” [7]. AEFIs can be divided into five broad categories [7, 8]:

1. Vaccine product-related: where a component of the vaccine is responsible for an adverse reaction
2. Vaccine quality-related: where the event is associated with a manufacturing process: for example, if a batch of vaccines becomes contaminated or a manufacturer loads it into faulty syringes
3. Immunization error-related: where the reaction is due to inappropriate handling, prescription, or administration of the vaccine: for example, if it is injected into the wrong body part or the vaccine accidentally gets frozen during transportation
4. Immunization stress-related: where the adverse event is because of the fear of being injected. This can result in physical responses: such as fainting, dizziness, tingling in the hands or around the mouth, vomiting, or even convulsions
5. Coincidental: where an adverse event has no direct relationship with the vaccine or any of the above, but it occurs soon after vaccination and hence may be attributed to it nonetheless

Adverse Event of Special Interest (AESI) is a preidentified and predefined medically significant event that has the potential to be causally associated with a vaccine product that needs to be carefully monitored and confirmed by further specific studies [9]. AESI encompasses serious reactions as well as severe yet rarely life-threatening or long-lasting problems such as allergic reactions or seizures [10]. One of the uncommon yet serious AEFIs, anaphylaxis is an IgE-mediated Type I Hypersensitivity reaction, which has been reported in one vaccine dose per million. Such allergic reactions may be due to active ingredients (a viral or microbial component in the case of the vaccine) or excipients used in the vaccine formulation such as preservatives, diluents, and buffers [10].

Through this article, we aim to review AEFI associated with currently available COVID-19 vaccines with the prime focus of narrating probable AEFI and assisting in developing an appropriate benefit-risk profile of the vaccines. [11].

## 2. Methods

To access the literature, search engines, such as Google Scholar, and databases such as PubMed and Cochrane review, were utilized. Meanwhile, official websites, reports of the WHO, Global Alliance for Vaccine Initiative (GAVI), Food and Drug Authority (FDA), and Center for Disease Control (CDC) were searched to access relevant content. The first article was searched in March 2021, and the literature search was carried out till July 2021. All the relevant articles found were organized using the reference manager Zotero 5.0.96.2.

Articles of interest were searched using Boolean operators. Each synonymous word was separated by a Boolean operator, “OR,” phrases were enclosed within quotation marks, and groups of synonymous words were enclosed within brackets. Each synonymous group of two or more different words was interlinked with the operator “AND.” For an extensive search in PubMed, the Medical Subject Heading (MeSH) database was used. For this review, we have considered reports from the WHO, government authorities, professional societies, observational studies, pharmacovigilance reports, case studies, and more than 90 pieces of published literature in English. These reports of AEFI associated with COVID-19 vaccines were extensively studied to extricate major conclusions. The keywords used for the literature search were “AEFI,” “adverse effect,” “pharmacovigilance,” “COVID-19 vaccine,” or any combination of these terms.

## 3. Findings

For ease of understanding this paper, we have classified COVID-19 vaccines in the following categories [12].

### 3.1. mRNA Vaccines

#### 3.1.1. Pfizer-BioNTech COVID-19 Vaccine (BNT162b2)

The most common adverse effects following the vaccination are flu-like symptoms such as soreness, fatigue, myalgia, headache, chills, fever, joint pain, nausea, muscle spasm, sweating, dizziness, flushing, feelings of relief, brain fogging, anorexia, localized swelling, decreased sleep quality, itching, tingling, diarrhea, nasal stuffiness, and palpitations [13–16]. While severe reactions, such as severe persistent lymphadenopathy or injection site pruritus lasting more than a week and pain (excluding headache, muscle, and joint pain) are not uncommon, effects like Bell's palsy are rare, with a frequency ranging from 1/10,000 to 1/1,000 [13]. The common adverse effects were more pronounced with the second dose, especially in the younger age group (below 45 years of age) and female population [13, 14, 17, 18]. Systemic side effects were reported by 13.5% and 22.0% of individuals after the first and second doses of the vaccine, respectively. Similarly, local and systemic adverse effects were found to be higher in individuals with a history of past infection with SARS-CoV-2 [16]. In addition, according to a randomized, cross-sectional study carried out among 803 healthcare workers, 103 (12.83%) temporarily had a problem doing their daily work, 99 (12.33%) took leave from work, 5 (0.62%) had to reach out to an outpatient service, and 2 (0.25%) needed hospitalization [19]. The CDC identified that among 1,893,360 recipients of the first dose of the Pfizer-BioNTech COVID-19 vaccine, 83 (0.004%) people reported nonanaphylaxis allergic reactions, whereas 21 (0.001%) people had anaphylactic reactions. Out of 21 recipients, 17 had a prior history of allergy to food, drugs, or vaccines such as the ARV and influenza vaccines [20].

#### 3.1.2. Moderna COVID-19 Vaccine (mRNA-1273)

Since Moderna is also an mRNA vaccine, the usual nonserious adverse effects are similar to those of Pfizer-BioNTech, with fatigue being the most common. The adverse effects of the Moderna vaccine were also found to be more intensified postsecond dose [14, 17]. In a study of 4,041,396 recipients of the first dose of the Moderna vaccine, 43 (0.001%) reported nonanaphylaxis allergic reactions, whereas 10 (0.0002%) females had anaphylaxis reactions, with a median time of 30 minutes from receiving the vaccine to the onset of reaction. Out of ten, five individuals had a history of allergy to substances like penicillin, intravenous contrast, and iodine [21]. Sore arm, myalgia, joint pain, nausea, confusion/brain fogging were some of the common adverse effects seen among the vaccine recipients of the United States [22].

### 3.2. Viral Vector Vaccines

#### 3.2.1. Oxford-AstraZeneca/Covishield COVID-19 Vaccine (ChAdOx1 nCoV-19)

The common adverse effects usually seen postvaccination with the Oxford/AstraZeneca COVID-19 vaccine are injection site pain, feverish feeling, muscle ache, and headache. These reactions were found to be less prevalent in recipients above 70 years of age as compared to those below 55 years of age [23]. About 33·7% and 58.7% of vaccine recipients developed systemic and local adverse effects, respectively, after the first dose of the vaccine [16].

Sah et al. reported that the recipients in Nepal developed mild headache and dizziness within 30 minutes of getting the first dose of ChAdOx1 nCoV-19 (Covishield): a formulation of the Oxford/AstraZeneca COVID-19 vaccine manufactured by Serum Institute of India Private Limited. Some of the vaccine recipients complained of irritability four hours postvaccination, whereas others complained of myalgia, nausea, tenderness at the site of injection, and fever with chills after 6-12 hours of vaccination, which were resolved with paracetamol intake. On the second to third day, the symptoms resolved partially [24].

Shrestha et al. from Nepal reported that apart from common AEFI, three severe AEFI were reported. The first case had abdominal cramps, loose stools, postural drop in blood pressure, and syncopal attack; the second one with abdominal cramps and postural drop in blood pressure; and the third one with urticaria and an episode of syncope [25]. Adhikari et al. reported injection site-related side effects as the most common AEFI, more prevalent in the age group below 30 years, with a *p* value of 0.007 (significant at *p* < 0.05) [26]. Interestingly, Madhi et al. have described the only serious adverse events observed in the recipients of the Oxford AstraZeneca COVID-19 vaccine as a fever above 40 degrees Celsius, which subsided within 24 hours [27].

#### 3.2.2. Janssen COVID-19 Vaccine (Ad26.COV2-S [Recombinant])

Pain at the injection site, headache, fatigue, muscle ache, and nausea are the common adverse effects reported postvaccination of the Janssen COVID-19 vaccine, which are self-limiting within a day or two [28]. In the mass vaccination of Janssen carried out in the US, out of 8,624 recipients, 64 (0.74%) cases of clusters of anxiety associated with tachycardia, hyperventilation, dyspnea, chest pain, paresthesia, light-headedness, hypotension, headache, pallor. Along with these, 17 (0.20%) cases of syncope have been reported [29]. Six suspected cases of clotting disorder were reported after the vaccination of the Janssen COVID-19 vaccine among seven million recipients, with the cause still under investigation [30].

#### 3.2.3. Gamaleya-Sputnik V COVID-19 Vaccine

The common side effects postvaccination include flu-like syndrome characterized by chills, fever, arthralgia, myalgia, asthenia, general discomfort, headache, and local reactions like injection site tenderness, hyperemia, and swelling [31]. The AEFIs were more common in people below 55 years of age (72.8% vs. 32%; hazard risk = 2.66) and in females (65.4% vs. 50%; hazard risk = 1.38). AEFI seemed to be more intense with the second dose as compared to the first [32, 33]. No serious adverse events were reported from phase I/II of the safety and immunogenicity study of the Sputnik V [34].

### 3.3. Inactivated Vaccines

Verocell, CoronaVac, and Covaxin are the inactivated vaccines being implemented in various nations. According to a study conducted in China, the prevalence of adverse effects in health care workers post-vaccination was 15.6% and 14.6% after the first and second dose, respectively. The most common is pain at the injection site, followed by fatigue, muscle pain, and headache [35]. Two cases of multiple sclerosis and Grade III emesis after vaccine uptake were also reported, both of which required hospitalization [36].

#### 3.3.1. Sinopharm-Verocell COVID-19 Vaccine

The most common local AEFI is pain at the injection site, while systemic AEFI are headache, fever, fatigue, myalgia, arthralgia, cough, dyspnea, nausea, diarrhea, and pruritus [37]. Aryal et al. from Nepal described mild to moderate AEFIs with the Sinopharm-Verocell COVID-19 vaccine. AEFIs were more common after taking the first dose of the vaccine compared to the second dose. No serious adverse events have been reported [38].

#### 3.3.2. Sinovac-CoronaVac COVID-19 Vaccine

A study by Riad et al. had reported the most common adverse effects postvaccination as pain at the injection site, fatigue, headache, myalgia, and arthralgia with a higher incidence of symptoms in females at *p* < 0.001 [39]. Some of the observed AEFIs with the vaccine were a case of serious hypersensitivity reaction with urticaria 48 hours after the first dose [40] and three cases of subacute thyroiditis postimmunization [41].

#### 3.3.3. Covaxin COVID-19 Vaccine

Following the administration of Covaxin, the most common adverse effects reported are pain at the injection site, headache, fatigue, fever, nausea, and vomiting [42]. No severe adverse effects have been reported so far [43].

## 4. Comparison of AEFI of Available COVID-19 Vaccines

### 4.1. Pfizer vs. Moderna COVID-19 Vaccines

A comparative study between Pfizer-BioNTech and Moderna COVID-19 vaccines concluded that both of them were responsible for causing adverse effects. However, the Moderna vaccine was likely to cause more adverse effects such as facial swelling and Bell's palsy, especially after the second dose [44, 45]. In another report by the Vaccine Adverse Event Reporting System (VAERS), the incidence of anaphylactic reactions in Moderna vaccine and Pfizer-BioNTech vaccine was 3/1,000,000 and 5/1,000,000, respectively [46].

### 4.2. Pfizer-BioNTech vs. Oxford-AstraZeneca Vaccines

In a study among healthcare workers in South Korea, the overall adverse reaction rate was 93% in the Pfizer-BioNTech group and 80% in the Oxford-AstraZeneca group (*p* < 0.001). Systemic reactions like fever, chills, muscle ache, joint pain, headache, dizziness, and fatigue were higher by 30% or more in the Oxford-AstraZeneca group compared with the Pfizer-BioNTech group. Similarly, neurological manifestations and allergy-like reactions were significantly more common in the Oxford-AstraZeneca group (*p* < 0.001) [47]. The incidence of rare anaphylaxis was associated with 0.63% of the recipients of Pfizer-BioNTech COVID-19 vaccines, whereas that with Oxford AstraZeneca COVID-19 vaccine was 0.3%, with the majority of it belonging to hemolytic anemia [48].

### 4.3. Pfizer-BioNTech vs. Moderna vs. Oxford-AstraZeneca Vaccines

From the study by Public Health Ontario, Canada, 5,140 (0.045%) AEFIs were observed out of a total of 11,212,134 vaccine recipients. Among these recipients, 207 (0.002%) had serious AEFI; 102 (49.28%) out of 207 were Pfizer-BioNTech COVID-19 vaccine recipients, 31 (18.84%) were Moderna recipients, and the remaining 74 (35.75%) were from the Oxford-AstraZeneca cohort [6]. The local and systemic effects seem to be more prevalent in mRNA (84.2%, 54.9%) and adenovirus vector vaccines (88%, 86%) as compared to inactivated vaccines (12%-18%, 4%-18%) [49].

## 5. System-Based AEFI

### 5.1. AEFI Related to Neurological Complications

Headache, dizziness, paresthesia, and muscle spasms are minor neurological AEFI associated with COVID-19 vaccination. However, minor cases of tremors, diplopia, tinnitus, dysphonia, seizures, and reactivation of the Herpes zoster have also been evident [50]. According to CDC's VAERS, 17 cases of stroke, 32 cases of Guillain-Barré syndrome, 190 cases of facial palsy, 6 cases of disseminated encephalomyelitis, and 9 cases of transverse myelitis were reported following Pfizer-BioNTech, Moderna, and Johnson and Johnson's COVID-19 vaccination [51].

A study conducted in Mexico by Garcia-Grimshaw et al. found that, of all 6536 AEFI, 4258 (65.1%) were related to mild neurologic manifestations such as headache, transient sensory symptoms, and weakness, while 17 (0.26%) cases showed AEFI related to serious neurological adverse events. The study concluded the vaccine's benefits outweigh the risk and that is why it was considered safe [52]. There has been one reported case of myelitis in India associated with the Oxford-AstraZeneca Covishield vaccine in a 36-year-old man on the 8^th^ day postvaccination [53]. Likewise, three cases (1.71%) of transverse myelitis (out of 175 serious adverse events) have been reported following the Oxford-AstraZeneca Covishield vaccination, of which one is after the second dose of the vaccine [54].

Several cases of facial nerve palsy have been reported post-Pfizer-BioNTech vaccination similar to that observed in influenza, Hepatitis B, polio, and DPT immunization. This is most likely caused by additive adjuvants that elicit an immunomodulatory response [55]. Overall, the evaluation of the preliminary results for various COVID-19 vaccines showed that neurological effects due to the vaccine are rare. However, the vaccine needs long-term monitoring to fully understand if the vaccine triggers any neurological issues [56].

### 5.2. AEFI Related to Cardiovascular and Hematological Complications

Oxford-AstraZeneca COVID-19 vaccines have shown a few cases of blood clotting disorders [57]. A 69-year-old man complained of reddish bruises on his wrist after the first dose of the Pfizer-BioNTech COVID-19 vaccine. The lab reports showed the prolongation of activated partial thromboplastin time and the presence of a factor VIII inhibitor. Few reports are available that Acquired Hemophilia A (AHA) is plausible with the use of vaccines in general or even with COVID-19 vaccines [58].

Likewise, a single case (0.0023%) of paroxysmal ventricular arrhythmia was identified among the 43,252 participants of a trial who received a single dose of Pfizer-BioNTech COVID-19 vaccine [59]. Palpitations (35, 8.1%), blood pressure changes (8, 1.85%), chest pain (8, 1.85%), and syncope (4, 0.93%) are common cardiovascular effects seen among Moderna recipients [22].

An 82-year-old woman appeared with a petechial rash in her lower extremities 10 hours post-CoronaVac vaccination was reported [60]. Likewise, a 22-year-old apparently healthy young male presented with widespread petechia and gum bleeding after receiving the Pfizer-BioNTech COVID-19 vaccine. The lab test showed a platelet count of 2 X 10^9^/L, which was diagnosed as severe thrombocytopenia [61]. Twenty cases of thrombocytopenia were hospitalized following Moderna and Pfizer vaccination; out of which, 17 had no prior history of bleeding disorder as reported by CDC, FDA, Department of Health and Human Service (HHS), VAERS [62]. The incidence of vaccine-induced prothrombotic immune thrombocytopenia ranges from 1/26,000 to 1/127,000 doses of ChAdOx1 nCoV-19 AstraZeneca/Covishield vaccine [63].

A case of central venous sinus thrombosis associated with thrombocytopenia was reported in a 50-year-old Caucasian man, 10 days after taking the first dose of the Oxford-AstraZeneca vaccine. Since the COVID-19 infection itself is associated with hypercoagulability, such conditions of thromboembolism cannot be neglected [64]. A reported event of acute right calf pain after 48 hours of the second dose of Pfizer-BioNTech COVID-19 vaccination was available. Color Doppler revealed deep vein thrombosis extending from the peroneal vein to the popliteal vein in the patient [65].

Various European countries like Denmark, Austria, Norway, and Italy halted the use of the Oxford AstraZeneca COVID-19 vaccine from the 11^th^ of March 2021, as multiple thrombosis and pulmonary embolism were observed after the first dose of the vaccine [66]. Among 54,571 adverse reactions post-Oxford AstraZeneca COVID-19 vaccination in the EudraVigilance database, 28 of these reactions were associated with thrombotic adverse effects, out of which three fatalities were related to pulmonary embolism and one to thrombosis. The incidence of such events seemed to be almost double in females [67]. In addition, 11 patients who had taken the AstraZeneca COVID-19 vaccine from Germany and Austria, presented with one or more thrombotic events: 9 had cerebral venous thrombosis, 3 had splanchnic venous thrombosis, 3 had pulmonary embolism, and 4 had other thromboses. Six of these patients died, and five had disseminated intravascular coagulation [68]. The exact mechanism of this significant incidence in females is not well understood, but it has been postulated that high levels of estradiol are associated with thrombotic events [69]. Meanwhile, the risk of cerebral venous thrombosis is 8 times higher in the population with COVID-19 history as compared to Oxford Astrazeneca COVID-19 vaccine recipients [68].

The Russian Gamaleya Center has stated, “a comprehensive analysis of adverse events during clinical trials and throughout mass vaccinations with the Sputnik V vaccine showed no cases of cerebral venous sinus thrombosis” [69]. However, the occurrence of immune thrombocytopenic purpura (ITP) is found to be 3.3 per 1,00,000 annually. The cases of ITP after the vaccine might be coincidental as well [70]. A wealth of studies have demonstrated the association between ITP and influenza vaccines, so this aspect cannot be completely overlooked [58].

According to Vigibase, 214 reports of COVID-19 vaccine-related myocarditis have been reported so far. Myocarditis was observed more in males, with a median age of 35 years, within a median of 3 days after taking the last dose of either the Pfizer or Moderna vaccine. Enough data was available to support the evidence that 23 cases were definite, 16 were probable, and 46 were possible myocarditis associated with the vaccine [71].

A pool analysis of case studies and case series [72] showed that 15 patients exhibited myocarditis following COVID-19 vaccination. More than 90% of these patients were male and had a median age of 28 years. Sixty percent of the cases were associated with Pfizer-BioNTech, 33% with Moderna and 7% with Jansen vaccine. All the cases related to Moderna vaccine occurred following the second dose of the vaccine, while 66.7% of the post Pfizer vaccination cases were observed after the second dose. From the overall analysis, the concluding points are as follows:

- Mostly healthy, young men are affected after the second dose of the vaccine
- AEFI is mostly associated with the mRNA vaccine
- All cases returned to good health without loss of cardiac function

### 5.3. AEFI Associated with Orofacial Manifestations

A study was carried out to study orofacial adverse effects in Pfizer-BioNTech and Moderna COVID-19 vaccine recipients in North America (the USA and Canada) and Europe (UK and EU). Heterogeneity was observed in orofacial adverse effects between North American and European vaccine recipients. Swelling of the lips, face, or tongue associated with anaphylaxis was common among North Americans, whereas acute facial peripheral paralysis (Bell's palsy) was more common among Europeans. The incidence of acute facial paralysis was greater in people with a history of injection of dermatological fillers [73].

### 5.4. AEFI Associated with Dermatological Manifestations

There are reports of cutaneous adverse effects similar to acute generalized exanthematous pustulosis and drug reaction with eosinophilia and systemic symptoms (AGEP-DRESS) overlap and morbilliform, urticarial, petechial, varicelliform, vasculopathy, and chilblain-like eruptions after Janssen COVID-19 vaccines [71, 72]. On the other hand, a 60-year-old man, a known case of hypertension and Type II diabetes mellitus, presented with fluid-filled lesions over the thigh four days after the Covaxin COVID-19 vaccine, which was later on diagnosed as herpes zoster shingles [74]. A similar clinical presentation was reported in a 78-year-old man with a history of multiple cardiovascular comorbidities and bladder cancer. He was consulted for erythematous, painful, and pruritic lesions on his chest, 5 days after taking the inactivated COVID-19 vaccine, which was also diagnosed as herpes zoster shingles [75].

A severely painful, unilateral dermatomal herpetiform eruption was observed in a 77-year-old man two days after receiving the first dose of the Moderna COVID-19 vaccine. Likewise, another case of painful, erythematous, and clustered skin eruptions was observed in a 65-year-old man after the second dose of Pfizer's vaccine who had a history of an episode of shingles 35 years ago. Twenty such cases of herpes have been reported in Las Vegas among Pfizer-BioNTech and Moderna vaccine recipients [76].

According to the FDA, the Moderna COVID-19 vaccine is capable of causing reactions like facial and lip swelling in patients with a history of dermal fillers [77]. Two cases of recipients developing acral chilblain-like lesions seven days postvaccination with CoronaVac have been reported [78].

For the purpose of better understanding the system-based AEFI of COVID-19 vaccines, the adverse effects are summarized in Table 1.

## 6. AEFI in Special Populations

### 6.1. AEFI in Pregnancy after COVID-19 Vaccination

Some studies have not only excluded pregnant women from immunization studies but also advised them to opt for contraception for weeks to months from the day of immunization [79]. Initially, pregnant and lactating mothers were excluded from the safety study of the COVID-19 vaccines. Therefore, the US FDA and the Advisory Committee on Immunization Practices stated that pregnant and lactating women were given an open option of whether to take vaccines [80].

Recently, the Royal College of Obstetricians and Gynecologists (RCOG) stated that minor adverse effects following vaccination are similar in pregnant and non-pregnant populations. However, pregnant women had a higher frequency of nausea and vomiting after the second dose of Pfizer-BioNTech and Moderna COVID-19 vaccines [81]. Similarly, the American College of Obstetricians and Gynecologists (ACOG) recommends COVID-19 vaccines for the pregnant population [82]. As per the CDC V-safe pregnancy registry, among 1,815 pregnant participants enrolled by February 19, 2021, in the vaccination program, 232 live births were delivered out of 275 completed pregnancies. Other cases included miscarriage (major), stillbirth, and ectopic pregnancies. [45].

With limited data so far, there is insufficient evidence to ascertain that COVID-19 vaccines have a beneficial or harmful action in pregnant women. Considering the risk-benefit ratio, different professional bodies such as RCOG and ACOG recommend the use of COVID-19 vaccines.

### 6.2. AEFI in Elderly after COVID-19 Vaccination

The importance of COVID-19 vaccination in senior citizens is vital since the risk of severe illness from COVID-19 increases with age. Thus, the CDC recommends COVID-19 vaccination among the elderly population. The proportion of minor side effects in the elderly were similar to those in other adult populations. The learning process on efficacy of COVID-19 vaccines in people with weakened immune systems is still ongoing [83].

## 7. Special Considerations

### 7.1. AEFI Associated with Excipients and Formulations

Allergic reactions might be elicited by active ingredients (a microbial or viral component) or by excipients of the vaccine [84]. Modified and truncated RNA traces might be present in Pfizer-BioNTech COVID-19 vaccines, and such aberrant proteins hold a minimal chance of eliciting allergic reactions [85]. Sputnik V COVID-19 vaccine is available in two forms: frozen and lyophilized, with frozen showing a high incidence of hyperthermia, headache, and muscle/joint pain. Despite this, there is no evidence of any serious adverse events [48]. The active constituent of the vaccine is not always responsible for eliciting adverse reactions. For instance, polyethylene glycol (PEG), one of the excipients of the Pfizer-BioNTech and Moderna COVID-19 vaccines, has been found to have induced IgE-mediated allergic reactions. Although Oxford AstraZeneca and Janssen COVID-19 vaccines have polysorbate 80, no allergic reactions have been noted to these vaccines. People allergic to PEG might also show cross-reactivity to PEG analogues (e.g. polysorbate), which should be systematically identified to prevent the chances of possible allergic reactions [17, 84–86]. Patients sensitive to latex may show anaphylactic reactions. Thus, even syringe plungers and vial stoppers may trigger such reactions [85].

### 7.2. AESI following COVID-19 Vaccines

From the study carried out across eight countries, the incidence of nonhemorrhagic stroke, acute myocardial infarction, and deep vein thrombosis were common in people above 85+ years of age. The incidence of acute myocardial infarction ranged from 1/10 to 1/100. [87].

### 7.3. AEFI Associated with Mortality

Out of 40,000 elderly patients, 30 very frail patients expired following Pfizer-BioNTech vaccination in Norway. This information questions the safety of the Pfizer-BioNTech COVID-19 vaccine in the elderly and critically ill patients [88]. Four deaths fulfilling provincial surveillance definition have been reported postvaccination in Ontario till June 12, 2021. However, only one death was reported due to vaccine-induced immune thrombotic thrombocytopenia (VITT) and thrombosis with thrombocytopenia syndrome (TTS). The remaining cases were stated as vaccine-unrelated [6]. A 68-year-old man who died following severe anaphylaxis was confirmed as the first mortality post-ChAdOx1 nCoV-19 (Covishield) vaccination by the government authorities of India [89].

## 8. Approach to AEFI of COVID-19 Vaccines

The Medicines and Healthcare Products Regulatory Agency (MHRA) stated that “any person with a history of anaphylaxis to a vaccine, medicine, or food should not receive the Pfizer/BioNTech vaccine” [90]. However, on December 30th, 2020, MHRA revised their statement that people showing such reactions have never been barred from receiving the vaccine [91]. Appropriate allergological evaluation helps in minimizing any immediate hypersensitivity reactions [92]. Hence, the sensible approach would be to enquire if the vaccine recipients have any prior history of allergy to food, medication, or vaccines. If there is any positive history, the susceptible people should be followed up by a specialist, so the vaccination can be conducted in a well-prepared environment [93]. Expanded skin testing procedures (skin pricking test and intradermal) with different dilutions of PEG to rule out PEG allergy is another way to avoid possible anaphylaxis [84]. Patients with negative skin tests should be kept under observation for 15 minutes after the vaccination, while those who test positive may require 30 minutes of observation to assess any adverse events [90, 93].

In people showing allergic reactions to PEG present in Pfizer-BioNTech and Moderna COVID-19 vaccines, cross-allergenicity to other PEG analogues must be tested. If found negative, the Oxford AstraZeneca COVID-19 vaccine can be considered an alternative [90]. However, the safer approach would be the use of neutral stabilizers such as polyvinylpyrrolidone or its derivatives that show an excellent safety record [85]. Emergency physicians should consider ITP due to vaccination among people who present with bleeding manifestations [91]. Meanwhile, dermatologists can participate actively in identifying dermatological manifestations postvaccination and contributing to tracking possible adverse reactions [94].

Due to the rapid development of COVID-19 vaccines, fear of their safety among healthcare workers and the public has led to vaccine hesitancy. Fear of COVID-19 vaccines and the vaccine hesitancy that follows can negatively impact regular immunizations. Open communication and public awareness regarding COVID-19 vaccines must be maintained to minimize public reluctance and improve vaccine uptake globally.

## 9. Conclusion

Allergic individuals cannot be excluded from vaccination. As AEFI with major case fatalities are very rare, vaccination should be encouraged since it helps prevent a potentially deadly illness. Moreover, health care personnel should clear up misconceptions regarding COVID-19 vaccines among the recipients. If any unfortunate event of anaphylaxis is observed, the patient must be transferred to receive appropriate medical care while the clinicians have to be vigilant to recognize, manage, and report the same.

## Figures and Tables

**Table 1:** System-wise AEFI of currently available COVID-19 vaccines.

System-wise AEFI vaccines	Occurrence of AEFI	General effects	Neurological manifestations	Cardiovascular manifestations	Hematological disorders	Dermatological manifestations	Gastrointestinal system
*mRNA vaccines*							
Pfizer-BioNTech vaccine	Common	Fever Fatigue Myalgia Injection site pain	Headache Confusion Seizures Paresthesia	Palpitations	Thrombocytopenia	Skin eruptions	Loose stools
	Uncommon		GBS Transverse myelitis Disseminated encephalomyelitis Bell's palsy Stroke^∗^	DVT^∗^ Ventricular arrhythmias			Anorexia
Moderna vaccine	Common	Fatigue Fever Myalgia Arthralgia Injection site pain	Headache Confusion	Palpitations	Thrombocytopenia	Herpetiform eruptions	Loose stools
	Uncommon		Bell's palsy Stroke^∗^	Blood pressure changes Syncope			
*Viral vector vaccines*							
Oxford-AstraZeneca/ChAdOx1 nCoV-19 (Covishield) vaccine	Common	Fever Myalgia Nausea Injection site pain	Headache			Urticaria	Loose stools Abdominal pain
	Uncommon		Transverse myelitis	Central venous sinus thrombosis Orthostatic hypotension Syncope Hemolytic anemia	Clotting disorders Pulmonary embolism Thrombocytopenia		
Janssen vaccine	Common	Fever Fatigue Myalgia Nausea Injection site pain	Headache Paresthesia		Clotting disorders	Skin eruptions	NA
	Uncommon		GBS	Hypotension Syncope		AGEP-DRESS	
Gamaleya-Sputnik V vaccine	Common	Fever Fatigue Myalgia Arthralgia Nausea Injection site pain	Headache	NA	NA	NA	NA
*Inactivated vaccines*							
Sinopharm-Verocell vaccine	Common	Injection site pain Fever Fatigue Myalgia Arthralgia Nausea Cough Dyspnea	Headache	NA	NA	Pruritis	Loose stools
Sinovac-CoronaVac vaccine	Common	Injection site pain Fever Fatigue Myalgia Arthralgia	Headache	NA	NA		NA
	Uncommon					Petechial rash Chilblain-like lesions	
Covaxin vaccine	Common	Injection site pain Fever Fatigue Nausea	Headache	NA	NA		Vomiting
	Uncommon					Fluid-filled lesions (herpes zoster)	

^∗^More common in the elderly population (above 85 years). AGEP-DRESS: acute generalized exanthematous pustulosis-drug reaction with eosinophilia and systemic symptoms; DVT: deep vein thrombosis; GBS: Guillain Barre syndrome; NA: not available.

## Data Availability

Data availability is not applicable.
